RETRACTED

# Temporal activation of anti- and pro-apoptotic factors in human gingival fibroblasts infected with the periodontal pathogen, *Porphyromonas gingivalis: *potential role of bacterial proteases in host signalling

**DOI:** 10.1186/1471-2180-6-26

**Published:** 2006-03-08

**Authors:** Sonya Urnowey, Toshihiro Ansai, Vira Bitko, Koji Nakayama, Tadamichi Takehara, Sailen Barik

**Affiliations:** 1 Department of Biochemistry and Molecular Biology, University of South Alabama, College of Medicine, 307 University Blvd., Mobile, Alabama 36688-0002, USA; 2 Department of Preventive Dentistry, Kyushu Dental College, Kitakyushu 803-8580, Japan; 3 Division of Microbiology and Oral Infection, Nagasaki University Graduate School of Biomedical Sciences, Sakamoto 1-7-1, Nagasaki 852-8588, Japan

## Abstract

**Background:**

*Porphyromonas gingivalis *is the foremost oral pathogen of adult periodontitis in humans. However, the mechanisms of bacterial invasion and the resultant destruction of the gingival tissue remain largely undefined.

**Results:**

We report host-*P. gingivalis *interactions in primary human gingival fibroblast (HGF) cells. Quantitative immunostaining revealed the need for a high multiplicity of infection for optimal infection. Early in infection (2–12 h), *P. gingivalis *activated the proinflammatory transcription factor NF-kappa B, partly via the PI3 kinase/AKT pathway. This was accompanied by the induction of cellular anti-apoptotic genes, including Bfl-1, Boo, Bcl-XL, Bcl2, Mcl-1, Bcl-w and Survivin. Late in infection (24–36 h) the anti-apoptotic genes largely shut down and the pro-apoptotic genes, including Nip3, Hrk, Bak, Bik, Bok, Bax, Bad, Bim and Moap-1, were activated. Apoptosis was characterized by nuclear DNA degradation and activation of caspases-3, -6, -7 and -9 via the intrinsic mitochondrial pathway. Use of inhibitors revealed an anti-apoptotic function of NF-kappa B and PI3 kinase in *P. gingivalis*-infected HGF cells. Use of a triple protease mutant *P. gingivalis *lacking three major gingipains (*rgpA rgpB kgp*) suggested a role of some or all these proteases in myriad aspects of bacteria-gingival interaction.

**Conclusion:**

The pathology of the gingival fibroblast in *P. gingivalis *infection is affected by a temporal shift from cellular survival response to apoptosis, regulated by a number of anti- and pro-apoptotic molecules. The gingipain group of proteases affects bacteria-host interactions and may directly promote apoptosis by intracellular proteolytic activation of caspase-3.

## Background

*Porphyromonas gingivalis*, a gram-negative anaerobe, is a major colonizer of gingival tissues, causing severe forms of adult periodontitis, in which the gingival fibroblast suffers extensive damage [1]. As replication inside mammalian cells is a common strategy adopted by many pathogenic bacteria, *P. gingivalis *infection has served as an important study model. A flurry of recent research has unraveled various pathways of interaction between oral cells and *P. gingivalis *[2]. Infection of various cell types by *P. gingivalis *activated cytokines and chemokines of potential importance in pathology, such as TNF-α, IL-1β, IL-6 and IL-8, the exact roles of which in adult periodontitis remain to be determined [3-7].

RETRACTED

*P. gingivalis *encodes a number of proteases, collectively known as 'gingipains', which have received considerable attention due to their multiplicity and potent activity [8,9]. The major members of this family include two Arg gingipains (RgpA and RgpB), and a Lys gingipain (Kgp) that are trypsin-like cysteine proteinases, specific for -Arg-Xaa- and -Lys-Xaa- peptide bonds, respectively. The gingipains were shown to regulate *P. gingivalis *adhesion and invasion positively as well as negatively depending on the cell type [10-12]. In a murine model of periodontitis, all contributed to virulence [13]. Recently, we and others have characterized a new protease of *P. gingivalis*, named endopeptidase O (PepO), and provided evidence for its importance in invasion and growth in human gum epithelial (HGE) and human lung epithelial (HEp-2) cells in culture [14,15].

A number of intracellular pathogens, including bacteria, viruses and parasites, either cause or suppress apoptosis of the infected mammalian cell by regulating a battery of pro- and anti-apoptotic genes [16-18]. Interestingly, various *P. gingivalis *protease preparations have been demonstrated to promote apoptosis when exogenously added to cells in culture [19-25]. The exact mechanism of this 'extrinsic' apoptosis is unknown but is believed to be triggered by the degradation of cell adhesion molecules such as neural cadherins and integrins by the proteases [25-28], which also causes detachment of the target cell from the tissue. It has been postulated that in periodontitis, apoptotic signals may overwhelm the normal anti-apoptotic forces that maintain periodontal vessels [29]. In contrast, *P. gingivalis *infection of human gingival epithelial (HGE) cells led to an anti-apoptotic response that paralleled the induction of mitochondrial anti-apoptotic Bcl-2 protein [30]. In a recent study externalization of membrane phosphotidylserine (PS) was noted immediately after *P. gingivalis *infection of HGE cells, suggesting an apoptosis-like response [31]. However, this was reversible, as the PS was internalized after 1 day of infection, and activation of the protein kinase AKT resulted in an anti-apoptotic response. Clearly, it is important to determine whether different gingival cell types respond differently to *P. gingivalis *and whether the gingipains play multiple regulatory roles in growth and pathogenesis.

RETRACTED

Although the fibroblast layer constitutes bulk of the gingival tissue, the molecular details of its interaction with *P. gingivalis *remain poorly understood. We decided to use primary human gingival fibroblast (HGF) cells in our studies for their obvious physiological relevance. In this communication, we analyze the status of programmed cell death or apoptosis in *P. gingivalis*-infected primary HGF cells and show that apoptosis is regulated in a stage-specific manner through the activation of an array of intracellular anti- and pro-apoptotic signalling molecules.

## Results

### Optimal infection of HGF cells by *P. gingivalis *requires a high m.o.i

Previous studies in which mammalian cells were infected with *P. gingivalis *in tissue culture typically used high multiplicities of infection (m.o.i.) – about 100–200 bacteria per human cell. It was not clear why such large number of bacteria were apparently needed for infection. A few studies that addressed the quantitative aspects of infection paid attention to the percentage of infecting bacterial cells but not to the percentage of infected mammalian cells. For example, in one study tests of m.o.i. 10, 100, 1000 and 10000 showed that the highest percentage of bacteria invaded HGE cells at 100 m.o.i. [32]. In another study using KB oral epidermoid carcinoma epithelial cells (likely to be HeLa cells), only about 2% bacteria attached to the cell monolayer at 50 m.o.i. of added *P. gingivalis *[11]. Single mutants lacking either protease RgpA or RgpB showed similar efficiency; however, when the *rgpA rgpB *double mutant was tested, about 60% bacteria attached to the epithelial cells. To explain this unexpected result, it was postulated that the Arg-gingipains may play a negative role in cell attachment by digesting the cellular receptors [11]. In all these experiments the percentage of infected KB cells remained undetermined. Role of KgP was also not tested. As attachment and invasion are the obligatory first steps in infection, we considered it important to determine the optimal efficiency of infection of HGF cells before proceeding to study the subsequent events.

To achieve this, we first quantified the efficiency of invasion. Washed wild type and triple gingipain mutant (*rgpA rgpB kgp*) *P. gingivalis *[33] were added to HGF monolayers and the infected HGF cells were counted by fluorescence staining with *P. gingivalis *antibody. A representative set of results (Fig. 1) show that there was a modest increase in the percentage of HGF cells infected with increasing m.o.i. Invasion reached a plateau at about 200 m.o.i., when roughly half of the cells were infected (Fig. 2). The triple protease mutant *P. gingivalis *fared worse, infecting only about a third of all cells at the same m.o.i. Although it is possible that some cells were infected at levels below the threshold of visible fluorescence, and therefore, were scored as uninfected, we can conclude that infection of HGF by *P. gingivalis *is a relatively inefficient process and that the Arg- and Lys-gingipains are not absolutely essential for invasion but improve the efficiency. Based on these findings (Fig. 2) and to achieve equal invasion we used an m.o.i. of 200 for the triple mutant and 80 for the wild type *P. gingivalis *in all subsequent experiments.

RETRACTED

Next, to determine the optimal time of release of progeny *P. gingivalis *from the infected cells, we assayed for bacterial colony forming units (cfu) in the HGF growth media at different times post-infection. This was done by plating serial dilutions of the media on agar plates as described in Materials and Methods. Maximal release of progeny bacteria occurred at 72 h post-infection coinciding with significant lysis of the monolayer (data not shown). Thus, we carried out all of our signalling experiments at earlier time points, usually not exceeding 48 h post-infection.

### *P. gingivalis *causes late apoptosis in infected HGF cells

At various times post-infection *P. gingivalis*-infected HGF cell monolayers were fixed and multiparametric staining including TUNEL staining for apoptosis was performed. Representative data (Fig. 3) show little apoptosis at early time point but significant apoptosis from 24 h onwards. Apoptosis was confirmed by propidium iodide-Annexin V staining (data not shown). The triple gingipain-mutant *P. gingivalis *also caused apoptosis but appeared to be slower and less effective.

As TUNEL is largely qualitative, we extended these studies with more detailed analyses (Fig. 4). A quantitative estimate of apoptotic nucleosome release was conducted, which supported the TUNEL kinetics and revealed that apoptosis by *P. gingivalis *is indeed a relatively late process in infection and that the mutant is less proficient in this regard (Fig. 4A). The DNA fragmentation paralleled activation of caspase-3, a major executioner caspase, using a synthetic fluorogenic substrate (Fig. 4B). We then investigated the activation of seven strategic caspases, including caspase-3, by immunoblot detection of their cleaved, active fragments, and the results (Fig. 4C) showed activation of caspase-6, caspase-7 and caspase-9 in addition to caspase-3, but not caspase-8, -10, or -12. Activation of caspases was found to occur late in infection, starting at around 24 h, coincident to apoptotic DNA damage. These results strongly suggested a role of specific caspases in *P. gingivalis*-induced apoptosis of HGF cells.

RETRACTED

For a direct measure of the intracellular caspase activity, we attempted to detect the breakdown products of αII-spectrin (also known as non-erythroid α-spectrin or α-fodrin). In apoptotic cells, the 240 kDa αII-spectrin undergoes a series of caspase-mediated cleavage to generate a major 120 kDa fragment, although a 150 kDa intermediate is sometimes detected as well [34]. Immunoblot analysis of *P. gingivalis*-infected HGF cell lysate (Fig. 4D) revealed the 120 kDa product, but only at late stages of infection, between 36 h and 48 h. The wild type *P. gingivalis *and the triple protease mutant produced essentially identical breakdown products that appeared much later in mutant-infected cells (48 h instead of 36 h). These results supported a caspase-induced breakdown of αII-spectrin and also matched the late-stage apoptosis and the slower kinetics of apoptosis by the mutant.

### *P. gingivalis *protease(s) directly cleave and activate procaspase-3 in vitro

Although the full impact of gingipains in host-bacterial interaction is still under investigation, their role in invasion is well-documented. As mentioned, exogenously added gingipains trigger extrinsic cell death, at least one mechanism of which involves the cleavage of external cell adhesion molecules such as cadherins and integrins [23,25]. Whether they have a role in the intrinsic pathways of apoptosis remains unknown. Although activated caspases are hallmark effectors of apoptosis, recent evidence suggests that non-caspase proteases such as cathepsins, calpains, granzymes, and the proteasome complex may have a direct caspase-like role in mediating apoptosis, but perhaps only in specific cell types or under specific signals [35,36]. Because *P. gingivalis *is a known producer of highly active proteases in the infected cells, it was worth testing whether these proteases might directly process and thereby activate an executioner caspase. To this end, we incubated purified recombinant procaspase-3 with *P. gingivalis *culture supernatant, and tested for cleavage. Results (Fig. 5A) show that the 34 kDa procaspase-3 was indeed cleaved to characteristic 17 kDa and 12 kDa fragments. The product sizes roughly matched with those produced by caspase-8-mediated cleavage of procaspase-3. Enzymatic activity of caspase-3 was confirmed by using the specific substrate peptide, DEVD (Fig. 5B). Similar amounts of culture supernatant made from the triple gingipain mutant exhibited little processing activity. Finally, the processing activity was destroyed by heat, in agreement with its protease nature. These results raise the interesting possibility that the Arg- and Lys-gingipains have the potential to directly contribute to apoptosis by activating intracellular caspase-3.

RETRACTED

### *P. gingivalis *infection of HGF cells leads to early activation of NF-kappa B

The proinflammatory transcription factor NF-kappa B (NF-κB) is generally responsible for suppression of apoptosis, although there are exceptions where it promotes apoptosis or has no apparent role in apoptosis [37]. In a number of obligatory parasites, infected cells are protected from apoptotic signals, mainly as a result of activation of NF-κB. In light of the apparent lag in apoptosis in the early stages of *P. gingivalis *infection it was important to determine whether NF-κB is activated in these cells. For a preliminary test, we first used an engineered HEK293 (hamster embryonic kidney fibroblasts) cell line that contained a chromosomal reporter luciferase gene under the control of NF-κB enhancers. Because of the convenience of luciferase assay, these cells are commonly used for rapid initial screening of NF-κB activating agents before detailed studies are done in more relevant cells. For example, we have shown previously that infection of these cells with respiratory syncytial virus leads to activation of NF-κB and hence, luciferase activity [38]. Conversely, inhibitors of NF-κB reduced the luciferase activity back to basal levels. As shown (Fig. 6A), a surge of luciferase activity was also detected at around 15 h following *P. gingivalis *infection of HEK293 cells. The levels gradually subsided from 24 h onward, suggesting loss of NF-κB activity. The gingipain-deficient strain also activated NF-κB albeit substantially weakly. SN50, a cell-permeable peptide inhibitor of NF-κB [39], strongly reduced luciferase activity, demonstrating specificity.

Having obtained positive results in luciferase assay, we proceeded to the physiologically relevant HGF cells and investigated NF-κB activation by direct measurement of the nuclear levels of the p65 subunit of NF-κB. In unstimulated cells, p65 is held back in the cytoplasm in complex with the inhibitors of κB, such as IκBα. Various signals including infection by many pathogens lead to the phosphorylation of IκBα via IκB kinase (IKK), followed by degradation of phospho-IκBα, allowing the nuclear import of p65 via its nuclear localization signal, where it activates transcription of NF-κB-dependent genes [40]. Thus, the appearance of NF-κB in the cell nucleus is indicative of its activation. It is seen (Fig. 6B) that *P. gingivalis *infection of HGF cells led to nuclear translocation of p65 early in infection that started to decline around 24 h. Phosphorylation of IκB was also detectable as early as 3 h p.i. (Fig. 6C), suggesting a correlation. A common upstream pathway leading to activation of NF-κB in many cells involves phosphoinositol-3 kinase, PI3K, and curiously, an inhibitor of PI3K (LY294002) inhibited IκB phosphorylation in these cells (Fig. 6C). This led us to study the potential role of PI3K in *P. gingivalis*-mediated activation of the NF-κB signalling, described next.

RETRACTED

### *P. gingivalis *infection activates the PI3K-AKT pathway

In mammalian cells, the PI3K/AKT pathway generally acts in a pro-survival, anti-apoptotic role [31,41]. A multitude of external stimuli activate intracellular PI3K that catalyzes the conversion of phosphatidylinositol 4,5-bisphosphate into the 3,4,5-triphosphate. The latter activates protein kinase PDK, which then phosphorylates AKT (also known as protein kinase B or PKB), thereby activating AKT. The activated AKT phosphorylates a large number of substrates such as Forkhead transcription factor (FKHR), IKK, Bad, caspase-9, and GSK-3. Together, these events inactivate the pro-apoptotic players such as Bad, and activate anti-apoptotic players such as NF-κB, leading to a net suppression of apoptosis.

We, therefore, determined the phosphorylation status of these signalling molecules in HGF cells during *P. gingivalis *growth using phosphospecific antibodies, and the results are presented in Fig. 7. It can be seen that all the major players of the pathway, namely PDK, AKT, Forkhead and GSK-3 were phosphorylated at comparable kinetics, early in infection. Total AKT protein levels did not change, confirming that the effect was truly on the phosphorylation status and not on protein synthesis. These anti-apoptotic phosphorylations occurred relatively early (≤ 6 h) and appeared to reach maximal levels by 6 h. In fact, at later times (between 12 and 24 h) phosphorylations reverted back to near pre-induction levels. The gingipain-deficient mutant also activated the same pathways with a similar kinetics. In all cases, the PI3K inhibitor, LY294002, abolished the phosphorylation, demonstrating that PI3K is indeed the most upstream kinase in this *P. gingivalis*-activated pathway. The same inhibitor also strongly inhibited the activation of NF-κB by *P. gingivalis *(Fig. 6A, striped bar), further supporting a role of PI3K in survival. Together, these results strongly support our premise that the early cellular response in *P. gingivalis*-infected HGF is anti-apoptotic whereas the late response is pro-apoptotic.

RETRACTED

### Temporal transcriptional induction of anti- and pro-apoptotic family genes by *P. gingivalis*

Studies over the last two decades have enlisted a large family of cellular genes that take part in either preventing or promoting apoptosis [42]. As the decision between cellular life and death is a net resultant of these two opposing forces, we decided to obtain a comprehensive view of expression of both families in *P. gingivalis*-infected HGF cells. The steady-state mRNA levels of major members of the two families were determined by reverse transcription and quantitative real-time PCR, and the results are presented in Fig. 8 as fold-induction over uninfected levels. The top two rows represent anti-apoptotic genes, and the rest are pro-apoptotic. The general trend that emerged from these results is that the two families were induced differently. The anti-apoptotic genes were induced early in infection, generally reaching their maximal levels by 12 h and then diminishing to variable extents over the rest of the infection period. The induction of a number of anti-apoptotic genes was sharply inhibited by the PI3K inhibitor, LY294002, as well as by the NF-κB inhibitor, SN50, further correlating the anti-apoptotic gene profile with the survival pathway. A representative example is Bfl1, the most robustly activated anti-apoptotic gene (Fig. 8, first box); both inhibitors caused 60–70% reduction of its induction. Similar inhibitory effect was also seen for three other genes tested, namely, Boo, Bcl-2, Survivin (data not shown).

In sharp contrast, the vast majority of the pro-apoptotic genes reached their maximum expression in later periods of infection, peaking between 24 and 36 h. Most were expressed poorly or not at all until about 12 h p.i. As in other pathways, the gingipain-deficient mutant activated these genes with similar overall kinetics. For the majority of the genes the mutant was weaker than the wild type although there were a few exceptions, such as the expression of Bcl-w, Bik, Bax, MOAP-1 was comparable in wild type and mutant-infected cells, and the induction of Bfl-1 and Bcl-XL expression was somewhat stronger in mutant-infected cells (Fig. 8). We carried out immunoblot (Western) analysis of selected representative proteins, namely Bcl-XL, Survivin, Bax and Bad, and the results essentially paralleled those of the transcript levels (data not shown). In conclusion, the general trend was that the expression of anti-apoptotic and pro-apoptotic genes was turned on early and late in infection, respectively, in a mutually exclusive chronological order.

## Discussion

One major finding in our study is the inefficient invasion by *P. gingivalis*, at least in cell culture, explaining the high m.o.i. traditionally used by all investigators. Although the exact mechanism needs further research, bacterial fimbriae, which are proteinaceous appendages extending from the bacterial cell surface, are known to play specific and important roles in bacterial adhesion and invasion, likely through an interaction with integrin and fibronectin of the host cell [43-45]. It is possible that these interactions are relatively inefficient and slow. Our results support the previous demonstration that Arg-gingipains enhance fimbriae-fibronectin binding, leading to the suggestion that the functional epitopes of cellular receptors of *P. gingivalis *are cryptic and that the Arg-gingipains expose them [46]. This is also consistent with our finding that the protease-deficient mutant *P. gingivalis *is a generally poor invader (Fig. 2).

RETRACTED

The second major finding here is that infection of primary gingival fibroblast cells by *P. gingivalis*, an important gum pathogen, leads to apoptosis, which may in part underlie the extensive tissue damage seen in gingivitis. Interestingly, early in infection, cellular anti-apoptotic genes are induced and postpone apoptosis; at later times, they give way to pro-apoptotic genes, and apoptosis ensues. As apoptosis is an exceedingly complex process involving a large variety of signalling molecules, we have focused our attention to selective major players.

The anti-apoptotic early phase in *P. gingivalis*-infected HGF cells is characterized by the activation of PI3K/AKT pathway. Our results (Fig. 7) strongly suggest that this pathway is largely responsible for the activation of pro-survival transcription factor NF-κB. The anti-apoptotic function(s) most likely facilitates *P. gingivalis *growth by thwarting premature dismantling of the host cell. The response of HGF and HGE cells to *P. gingivalis *infection, therefore, has interesting similarities and differences. Like HGF cells, infection of HGE cells resulted in suppression of apoptosis, which required phosphorylation-mediated activation of AKT and was inhibited by LY294002 [31]. However, HGF cells eventually became apoptotic whereas HGE cells appeared to remain anti-apoptotic. Thus, the fibroblasts and epithelial cells of the same tissue may differently regulate the apoptotic modulators, the mechanism of which must await further study.

Caspases are a class of cysteine proteases that includes several representatives involved in apoptosis [42]. They are activated via a proteolytic cascade, cleaving and activating other caspases, eventually degrading downstream targets and promoting cell death (Fig. 9). The main "initiator" caspases at the upper end of the cascade are caspase-8 and caspase-9. Caspase-8 is activated in response to death receptors (such as Fas) whereas caspase-9 is activated by the release of cytochrome c via the intrinsic mitochondrial stress pathway. Activation of caspase-9 but not caspase-8 in *P. gingivalis*-infected HGF cells (Fig. 4) strongly points to the activation of the mitochondrial pathway. Clearly, caspase-9 then activates the downstream "executioner" caspases, namely caspase-3, -6 and -7. Spectrin fragments serve to distinguish between caspase-3 and calpain; while caspase-3 cleavage generates the 120 kDa fragment calpain produces 150 and 145 kDa fragments [34,47]. Our results, therefore, confirms caspase-3 activation (Fig. 4) and rules out a role of calpain in *P. gingivalis*-mediated apoptosis. A novel apoptotic pathway has been discovered recently, in which an endoplasmic reticulum (ER) resident caspase, namely caspase-12, is activated by ER stress that may be triggered by heavy traffic of glycoproteins through the ER. For example, we have shown that infection by respiratory syncytial virus, a cytoplasmic RNA virus expressing three glycoproteins that traffic through the ER, causes late apoptosis in lung epithelial cells by activating ER-stress and caspase-12 [16]. Together, results presented here suggest that *P. gingivalis *activates apoptosis through the mitochondrial pathway and not the ER or Fas pathway.

RETRACTED

Based on these findings, we present a working hypothesis of *P. gingivalis*-activated apoptosis in HGF cells in Fig. 9. We emphasize that it is not a comprehensive list and that we have provided experimental evidence only for the key players in each major branch. In the anti-apoptotic early phase, we have demonstrated activation of PDK, AKT / PKB, the AKT substrates (GSK-3 and FKHR) and the IKK substrate (IκB-α) (Fig. 7). The involvement of PI3K and NF-κB was also uncovered by the use of specific inhibitors. Transcriptional activation of a battery of anti-apoptotic genes is also indicated (Figs. 8, 9), which was abrogated by inhibitors of either PI3K or NF-κB. The pro-survival role of the PI3K/NF-κB pathway is explained by the recent demonstrations that transcription of these anti-apoptotic genes is NF-κB-dependent [48].

In the pro-apoptotic late phase of infection, we surmise a major role for the mitochondria. One of the best characterized mechanisms used by mitochondria to induce cell death is the release of pro-apoptotic proteins into the cytosol [49]. Cytochrome c, the first molecule shown to be released, complexes with apoptosis protease-activating factor 1 (Apaf-1) and exposes domains of Apaf-1 that activate caspase-9. A proteolytic cascade ensues that eventually activates caspases-3, -7 and -6 (Fig. 9), and our results show activation of all these caspases (Fig. 4). Nucleosomal DNA degradation (Figs. 3, 4) suggested the activation of DNA-fragmentation factor (DFF), although the involvement of AIF and endonuclease G, released from stressed mitochondria (Fig. 9) cannot be ruled out. Most importantly, the kinetics of activation of these proteins was in accord with the shift from an anti- to a pro-apoptotic response.

RETRACTED

Further evidence for the shift came from transcriptional data of anti- and pro-apoptotic genes. The mitochondrial Bcl-2 family [49] comprises of both kinds, such as the anti-apoptotic members Bcl-2, Bcl-XL, Bcl-w, Mcl-1 and the pro-apoptotic members Bax, Bak, Bok, Bid, Bad, Puma, Bmf, Bim, Bok, Noxa and Hrk/DP5. Some of the most highly activated genes in Fig. 8 indeed belong to these two families and their functions match with the temporal shift from survival to death. However, the relative contribution of each of these proteins in regulating apoptosis is currently unknown.

The direct processing of procaspase-3 by *P. gingivalis *protease(s) (Fig. 5) adds a novel dimension to 'intrinsic' apoptosis by bacteria. Interestingly, structural analysis of the catalytic subunit of Rgp revealed a caspase-like fold, suggesting a common ancestor [50]. Moreover, homology mapping suggested that a single protease clan, named CD [51] or the caspase-hemoglobinase fold [52], encompasses gingipains and caspases as well as bacterial clostripain and legumains (processing proteases) [53,54]. As the processing by gingipains generated enzymatically active caspase-3 (Fig. 5), it is reasonable to conjecture that the cleavage occurred at or close to the natural processing site. The processing defect of the *rgpA rgpB kgp *mutant suggests that the cleaved peptide bond would be next to either an Arg or a Lys. The natural processing in procasapse-3 is known to occur next to the Asp^175^, shown here in bold within the substrate motif IETD: CR^164^GTELDCGIET**D**^175^SGVDDDMACHK^186^. We noticed Arg^164 ^and Lys^186 ^nearby (as underlined in the sequence), 11 residues upstream and downstream of the Asp^175^, respectively. We speculate that one or more of the gingipains cleave the procasapse-3 at either or both of these sites to produce the activated caspase-3. This is currently being tested. The physiological significance of this activation also needs to be resolved. It is possible that the anti-apoptotic functions antagonize this activation and prevents it from happening too early in infection. Moreover, note that the mutant strain is not completely defective in activating apoptosis and caspase-3 in HGF cells (Fig. 4). Thus, the three gingipains, although not absolutely essential, seem to be needed for optimal apoptotic response.

RETRACTED

We note here that the gingipains may be partially sequestered by serum proteins; human [55] and bovine (our unpublished results) serum albumin, for example, are excellent substrates for gingipains. It is also possible that serum will contain unidentified inhibitors of gingipains [55]. On the other hand, the presence of serum likely approximates the physiological infection of the gum and provides an optimal nutrient level for intracellular replication of the bacteria. For the best compromise, therefore, we allowed the bacteria to invade initially for 90 min in the absence of serum, and then replaced it with serum-supplemented medium for further growth (Materials and Methods).

It is tempting to speculate that the delayed apoptosis of the host cell most likely allows *P. gingivalis *extra time to replicate intracellularly to a higher yield and at the same time offers early protection to the infected cells against cytotoxic mediators of the host immune system. An extended period of nuclear DNA integrity may also allow the cell to transcriptionally activate genes that modulate immune or inflammatory response. Apoptosis then occurs at the late stage of infection when the replicated bacteria must destroy the host cell anyway in order to egress and infect neighboring cells for fresh nutrients and continued growth. Clearly, a detailed knowledge of how *P. gingivalis *regulates the balance between multiple apoptotic signalling molecules in chronological order will shed important light on the mechanism of tissue damage in gingivitis and may provide a pharmacological regimen to control the infection.

## Conclusion

*P. gingivalis *infection of human gingival epithelial cells initially triggers a survival response through the activation of PI3K/AKT pathway, resulting in the activation of NF-κB and a family of anti-apoptotic proteins. This likely allows optimal growth of the bacteria. At later stages of infection the anti-apoptotic proteins subside and pro-apoptotic ones are turned on, leading to apoptosis of the infected cell. Bacterial proteases of the gingipain family play important roles in various aspects of infection, including proteolytic activation of caspases by processing, which may directly contribute to the observed apoptosis. Thus, *P. gingivalis *and the host gingival cell interact via a variety of pathways that are relevant in the pathology and degradation of the gingiva.

## Materials and methods

### Materials

Antibodies against the following antigens were obtained from commercial sources: p65, Sp1 (Santa Cruz Biotechnology); phospho-AKT, caspases-3, -6, -7, -8, -9 (Cell Signaling Technology); caspase-10 (Oncogene); caspase-12 (Sigma); IκB-α (Biomol); nonerythroid alpha-spectrin (Chemicon International); Bcl-XL, Survivin, Bax and Bad (Sigma-Aldrich). Other phosphospecific antibodies were from New England Biolabs. The phosphatase inhibitor cocktail set II (final concentration of 1 M imidazole, 0.1 M sodium fluoride, 0.115 M sodium molybdate, 0.2 M sodium orthovanadate, and 0.4 M sodium tartrate) and the inhibitors LY294002, SN50 and staurosporine were from Calbiochem (San Diego, CA). "Complete protein inhibitor cocktail" was from Roche, one mini tablet of which was added per 10 ml of buffer (final concentration) as prescribed by the manufacturer.

RETRACTED

### Bacteria and culture conditions

Wild-type *P. gingivalis *(ATCC 33277) and the isogenic mutant strain (*rgpA rgpB kgp*) [33] were grown anaerobically (85% N_2_, 10% H_2_, and 5% CO_2_) at 37°C in brain-heart infusion broth supplemented with yeast extract (0.5%), hemin (5 μg/ml), and menadione (0.5 μg/ml), essentially as described [56]. Bacteria were grown to mid-log phase (A_600 _in the range of 0.6–0.8), harvested by centrifugation, washed with phosphate-buffered saline (PBS) and resuspended in DMEM supplemented with 2 mM L-glutamine. For each experiment the final concentration of the suspension was determined by measurement of A_600 _and appropriate dilutions were made to achieve the desired m.o.i. The bacterial number was confirmed retroactively by viable counting of colony forming units (cfu) on agar plates supplemented with hemin and menadione [32,56].

### Culture of HGF cells

Primary cultures of HGF cells were made from biopsies of healthy human gingival obtained from dental clinics. The tissues were washed several times in PBS and DMEM, then cut into small pieces and placed in a T-25 cm^2 ^flask with complete medium containing DMEM supplemented with 10% FBS, 2 mM L-glutamine, 2.5 μg/ml fungizone, and 5000 U/ml penicillin/ streptomycin. When ready for passage, the fibroblast cells were cultured as monolayers in the same complete media without fungizone at 37°C in a standard 5% CO_2 _incubator.

### Infection of HGF cells with *P. gingivalis*

HGF cells were used at 80 to 90% confluency for all experiments. Before infecting with *P. gingivalis*, the monolayers were washed three times with PBS. *P. gingivalis*, resuspended in DMEM without FBS or antibiotics, was added to the HGF monolayer at the desired m.o.i. and incubated for 90 min at 37°C in 5% CO_2_. The monolayer was then washed twice with PBS to remove unbound bacteria, DMEM supplemented 10% FBS and 2 mM L-glutamine was added, and growth continued at 37°C in 5% CO_2_.

RETRACTED

Assessment of bacterial invasion was done by an antibiotic protection assay essentially as described previously with minor changes [11,14,32]. HGF cells were first infected with washed *P. gingivalis *and external, nonadherent bacteria were removed as described above. The cultures were then incubated for an additional 2 h at 37°C in fresh medium containing 300 μg gentamicin and 200 μg of metronidazole per ml to kill the remaining extracellular bacteria [32]. We confirmed that the antibiotics did not affect the morphology of the HGF cells or alter their ability to exclude trypan blue. Following invasion, the HGF cells were fixed and stained as described below.

### Immunofluorescence studies and assays of cell death and NF-κB

For multiparametric staining, HGF cells were grown on coverslips in 6-well plates to 80–90% confluency. The cells were then infected with washed *P. gingivalis *as above. Coverslips were washed three times with PBS and fixed in 10% trichloroacetic acid for 20 min on ice. Successive washes were then performed with 70%, 90% and 100% ethanol, and finally with PBS containing 0.2% Triton X-100. The coverslips were incubated with a rabbit antibody against *P. gingivalis *Fim A and then with secondary mouse antibody (TRITC-conjugated). Finally, the coverslips are mounted on a slide with DAPI-DABCO solution and observed by fluorescence microscopy in an Olympus BMAX Epifluorescence microscope [16]

For routine detection of apoptosis, we used the DeadEnd Fluorometric TUNEL System (Promega) that measures apoptosis by the integrating fluorescein-12-dUTP at 3'-OH DNA ends of fragmented DNA of apoptotic cells. The fluorescein-12-dUTP-labeled DNA was visualized directly by fluorescence microscopy. Cells are grown to confluency on coverslips in 6-well plates and stained as per the manufacturer's instructions. Annexin V, conjugated with fluorescein isothiocyanate (FITC) (Sigma), was used to label phosphatidylserine on the apoptotic membrane surface, and propidium iodide (PI) to stain the nuclei (if necrotic).

Quantitative assay of apoptosis was performed with a new procedure termed "Cell Death Detection ELISA" (Roche) which involves photometric enzymatic immunoassay of mono- and oligo-nucleosomes in the cytoplasmic fraction of apoptotic cell lysates.

Luciferase reporter assay for NF-B was performed as described [38]. Briefly, cells in monolayer were transfected with pNFκB-Luc using Lipofectin^® ^(Gibco Life Technologies), and infected with washed *P. gingivalis *cells 24 hr later. When used, inhibitors were added at the same time as the bacteria. The cells were lysed at indicated times thereafter and cleared extracts subjected to luciferase assay in a Turners Design luminometer [38].

RETRACTED

### Data acquisition and analysis

In invasion assay as well as in apoptosis detection, the fluorescent HGF cells were visually counted using a subjective baseline that corresponded to uninfected controls. Changes were analyzed by one-way ANOVA and then by Student's t-test with Bonferroni correction. All numerical data were collected from at least three separate experiments. Results were expressed as mean ± SEM (error bars in graphs). Differences were considered to be significant at P < 0.05.

### Quantitative real-time PCR

HGF cells were grown in T-25 flasks and infected with wild-type and mutant *P. gingivalis *as described. At different time points, mRNA from infected cells was purified using a Trizol method (Ambion). First-strand cDNA was made using the GeneAmp RNA PCR Core kit (Perkin Elmer-Applied Biosystems). Primers were designed by the Beacon Designer software v 2.13 from Premier Biosoft essentially as described previously [57], and are listed in Table 1. Real Time PCR was performed on the iCycler iQ Quantitative PCR system from BioRad Laboratories (Hercules, CA) using the iQ Sybr Green SuperMix. Gene expression measurements were calculated using the manufacturer's software; GAPDH was used as an internal control.

### Immunoblot (Western) analysis

The infected monolayer and any control samples were washed twice in PBS containing the protease inhibitor cocktail described under Materials. When phosphoproteins were to be detected, all buffers additionally contained the phosphatase inhibitor cocktail. The cells were scraped off in PBS containing the inhibitors and centrifuged at 5,000 × g for 10 min to remove cell debris. The pellets were boiled in standard SDS sample buffer, and proteins separated by 12% SDS-PAGE and transferred to nitrocellulose [58]. Blots were probed with the appropriate antibody followed by corresponding secondary antibody coupled to horseradish peroxidase, and developed using the ECL kit (Pierce). The chemiluminescence was detected in LAS-1000 plus imaging system (Fuji Film).

For NF-κB, the infected monolayer in 6-well plates was washed twice with PBS containing the protease inhibitor cocktail. Fifty microliters lysis buffer (50 mM Tris-HCl [pH 8.0], 50 mM NaCl, 0.1 mM EDTA, 0.1% Tween 20, 1x protease inhibitor cocktail) was then added to the cells in each well. The cells were scraped in the buffer and centrifuged at 15,000 × g for 15 min at 4°C. The resulting supernatant was used as the cytosolic extract; the pellet was washed twice with the same buffer (5,000 × g for 10 min at 4°C) and used as the nuclear fraction.

RETRACTED

### Caspase cleavage and assay

Overnight grown *P. gingivalis *cells were collected by centrifugation at 10,000 × g and washed three times with PBS. Pellets were resuspended in DMEM (without serum or antibiotic) and incubated for 4 h anaerobically (85% N_2_, 10% H_2_, and 5% CO_2_) at 37°C. Supernatant was collected by centrifugation (14,000 × g) and protein concentration determined by Bradford assay (Bio-Rad).

To test for the cleavage activity, pre-determined amounts of the supernatant were incubated with 5 μg of purified procasapase-3 (Biomol) at 37°C in a 50 μl reaction in the following buffer: 50 mM Hepes (pH 7.5), 50 mM NaCl, 20% glycerol, 0.1% CHAPS, 1 mM DTT. The supernatant was substituted with purified caspase-8 (Biomol) in a positive control reaction and with same volume of buffer in a negative control. Portions of the reaction were analyzed by SDS-PAGE and immunoblot [57]. The rest of the reaction was assayed for caspase-3 activity using the colorimetric substrate, DEVD-*p*NA, which upon cleavage exhibits increased absorption at 405 nm (Calbiochem). Reactions were incubated at 30°C and followed with time in a spectrophotometer to ensure linearity.

## Authors' contributions

SU did the major experiments; TA performed initial assays of invasion in the SB laboratory; VB carried out additional invasion studies and caspase assays; KN constructed the mutant strains; TT offered expertise and guidance to TA; SB conceived and guided the project, and wrote the paper with help from SU. All authors read and approved the final manuscript.

## Figures and Tables

**Figure 1:** Infection of HGF cells by *P. gingivalis*. Wild type (WT) or triple gingipain mutant (MT) *P. gingivalis *was added to monolayers of HGF cells at the indicated bacteria-to-cell ratios (m.o.i). Only a few representative multiplicities are shown. Invasion was determined after killing of the external bacteria with antibiotics and staining the cells with DAPI (Blue) and *P. gingivalis *Fim A antibody (Pg; Red) as described under Experimental Procedures. Visually detectable red cells in the 'Pg' fields were counted in three independent observations and expressed as percentage of all the blue cells in the 'DAPI' fields.

**Figure 2:** Multiplicity-dependent increase of HGF invasion by *P. gingivalis*. Invasion results obtained by staining (from Fig. 1) are plotted here. Error bars from three experiments are shown.

**Figure 3:** Apoptosis in HGF cells by *P. gingivalis *infection. Infection of HGF monolayers and staining for all nuclei (DAPI, Blue) or only the apoptotic ones (TUNEL, Green) were carried out as described under Experimental Procedures. Cells were infected by wild type (WT) or the triple gingipain mutant (MT), and stained at the indicated time of infection (5 h, 24 h, 48 h). For positive control of apoptosis, uninfected HGF cells were treated with staurosporine for 5 h.

RETRACTED

**Figure 4:** Kinetics of apoptosis and caspase activation following *P. gingivalis *infection. HGF monolayers were infected with wild type (WT) or triple gingipain mutant *P. gingivalis *and harvested at indicated times for the following assays as described under Experimental Procedures. (A) DNA fragmentation assay using the "Cell Death Detection ELISA" (Roche); (B) Caspase-3 activity assay in cell lysates; (C) Immunoblot detection of activated (cleaved) caspases in HGF cells infected with WT, with Sp1 serving as a control for equal protein loading; note the absence of activated caspases-8, -10, -12. (D) Immunoblot detection of α-spectrin fragments in infected HGF cells; the full-length 240 kDa spectrin and the caspase-specific 120 kDa product bands are so marked. In A and B, the standard error bars are from three experiments.

**Figure 5:** Cleavage (A) and activation (B) of procaspase-3 by *P. gingivalis*-excreted gingipains. (A) Incubation of pure procaspase-3 with caspase-8 (4 or 8 ng) or culture supernatants ('sup') of wild type (WT) or triple gingipain mutant (MT) *P. gingivalis *(20 or 40 ng protein content, labeled over lanes) were done as described under Experimental Procedures. The products were analyzed by SDS-PAGE and silver-staining. The full-length procaspase-3 (34 kDa) and the processed active fragments (17 and 12 kDa) are marked by open and closed arrowheads, respectively. (B) Activity of the processed caspase-3 generated in Panel A was measured using a colorimetric peptide substrate described under Experimental Procedures. The enzymes used to cleave procsapase-3 are: 20 ng of wild type *P. gingivalis *sup (Triangle); 4 ng caspase-8 (Squares); 20 ng of gingipain mutant *P. gingivalis *sup (Open circles); 20 ng of wild type *P. gingivalis *sup, preheated at 65°C for 15 min (Diamonds); none (Closed circles). The error bars are derived from three independent experiments.

**Figure 6:** PI3K-dependent activation of NF-κB by *P. gingivalis*. (A) Activation of NF-κB-dependent luciferase in HEK cells. Monolayers were infected with wild type *P. gingivalis *in the presence of no drug (Open bars), 20 μM SN50 (Speckled bars), 20 μM LY294002 (Striped bar), or with the triple gingipain mutant (Closed bars), and luciferase assay carried out as described in Materials and Methods. Error bars represent average of three experiments. (B) Nuclear import of NF-κB p65 subunit. HGF cells were infected with *P. gingivalis *(wild type = WT; gingipain mutant = MT), and nuclear extracts (40 μg protein) of infected cells (or uninfected controls = U) were analyzed for p65 by immunoblot [54]. Sp1 serves as an unchanged control. (C) Phosphorylated IκB-α, an indicator of NF-κB activation, was detected by immunoblot of the total infected HGF cell extract using a specific antibody [54]. This phosphorylation was undetectable when 20 μM LY294002 (PI3K inhibitor) was included in the culture medium (+I).

RETRACTED

**Figure 7:** Activation of members of the PI3K/AKT pathway. HGF monolayer was infected with wild type *P. gingivalis *(WT) or its triple gingipain mutant (MT), and the infected cells grown in the presence (+I) or absence of 20 μM LY294002 (PI3K inhibitor). Total cell extracts (50 μg) were probed in immunoblot for the presence of total AKT or specific phosphorylated proteins of the AKT pathway as named. The two species of phospho-FKHR are indicated by closed circle and triangle. Note the early (6–12 h) activation of phosphorylation and its inhibition by the inhibitor.

**Figure 8:** Induction of apoptosis-related gene mRNAs in HGF cells infected with wild type *P. gingivalis *(Triangles) or its triple gingipain mutant (Circles). Total mRNA from infected cells at different times p.i. were subjected to quantitative Real Time RT-PCR as described under Materials and Methods, using primers described in Table 1. The relative amounts of RNA were expressed as the ratio of uninfected control value (fold induction). Each box represents a specific gene as named and its generally accepted nature as anti-apoptotic ('anti') or pro-apoptotic ('pro'). Each data point is derived from three independent infection experiments with the error bar as shown. Note the general trend of early activation of anti-apoptotic genes (upper rows) and late activation of the pro-apoptotic ones (lower rows). Treatment with LY294002 (Closed circles) and SN50 (Closed triangles) inhibited activation of anti-apoptotic genes, as exemplified by Bfl-1.

**Figure 9:** A working model for *P. gingivalis*-activated apoptosis in HGF cells. Note that this is a highly reductive and simplified model showing only the major signaling events and that the intermediate steps are mostly omitted for space (details in Results and Discussion). In general, the *P. gingivalis*-activated molecules shown in this paper are displayed more prominently. The ER stress and Fas pathways were not activated. Whether the gingipains activate caspase-3 *in vivo *remains a question. The box on the left lists the major anti-apoptotic molecules activated early in infection, and the box on the right shows the pro-apoptotic molecules activated later. The two sets of forces are mutually antagonistic and thus, the balance shifts from anti- to pro-apoptosis as infection progresses.

RETRACTED

**Table 1:** The apoptosis family genes and their PCR primers

Gene, Accession #	Sense	Antisense
Bfl-1, NM_004049	TTACAGGCTGGCTCAGGACT	CCCAGTTAATGATGCCGTCT
Boo, NM_020396	GAAGAAGTGGGGCTTCCAG	GAAAGGGGGTCCTGAAGAAG
Bcl-XL, NM_138578	GTAAACTGGGGTCGCATTGT	TGGATCCAAGGCTCTAGGTG
Bcl-2, NM_000633	ATGTGTGTGGAGAGCGTCAA	ACAGTTCCACAAAGGCATCC
Mcl-1, NM_021960	TAAGGACAAAACGGGACTGG	ACCAGCTCCTACTCCAGCAA
Survivin, NM_001168	GGACCACCGCATCTCTACAT	GACAGAAAGGAAAGCGCAAC
Bcl-w, NM_004050	GCTGAGGCAGAAGGGTTATG	CACCAGTGGTTCCATCTCCT
Nip3, NM_004052	CTGGACGGAGTAGCTCCAAG	TCTTCATGACGCTCGTGTTC
Hrk, NM_003806	CTAGGCGACGAGCTGCAC	ACAGCCAAGGCCAGTAGGT
Bak, NM_001188	TTTTCCGCAGCTACGTTTTT	GGTGGCAATCTTGGTGAAGT
Bik, NM_001197	TCTTGATGGAGACCCTCCTG	GTCCTCCATAGGGTCCAGGT
Bok, NM_032515	AGATCATGGACGCCTTTGAC	TCAGACTGCAGGGAGATGTG
Bax, NM_004324	TCTGACGGCAACTTCAACTG	CACTGTGACCTGCTCCAGAA
Bad, NM_004322	CGGAGGATGAGTGACGAGTT	CCACCAGGACTGGAAGACTC
Bim, NM_207003	TGGCAAAGCAACCTTCTGAT	TCTTGGGCGATCCATATCTC
Moap-1, NM_022151	CAGTGGGTGAGTTGAGCAGA	GAAACATCCAGCGTCCAAAT

The common names of the anti- and pro-apoptotic genes and their RefSeq accession numbers (GenBank) are shown here. The sense and antisense sequences correspond to the RT-PCR primers used for amplification of the transcripts by real-time PCR (Fig. 8). All sequences are written 5' to 3'.
